This article has been retracted.

# Glycolipid Metabolism Disorder in the Liver of Obese Mice Is Improved by TUDCA via the Restoration of Defective Hepatic Autophagy

**DOI:** 10.1155/2015/687938

**Published:** 2015-11-19

**Authors:** Qinyue Guo, Qindong Shi, Huixia Li, Jiali Liu, Shufang Wu, Hongzhi Sun, Bo Zhou

**Affiliations:** ^1^Critical Care Medicine, The First Affiliated Hospital of Medical School of Xi'an Jiaotong University, 277 Yanta West Street, Xi'an, Shaanxi 710061, China; ^2^Key Laboratory of Environment and Genes Related to Diseases, Medical School of Xi'an Jiaotong University, Xi'an, Shaanxi 710061, China; ^3^Center for Translational Medicine, The First Affiliated Hospital of Medical School of Xi'an Jiaotong University, 277 Yanta West Street, Xi'an, Shaanxi 710061, China; ^4^Department of Respiratory, The First Affiliated Hospital of Medical School of Xi'an Jiaotong University, 277 Yanta West Street, Xi'an, Shaanxi 710061, China

## Abstract

*Objective. *Tauroursodeoxycholic acid (TUDCA) has been considered an important regulator of energy metabolism in obesity. However, the mechanism underlying how TUDCA is involved in insulin resistance is not fully understood. We tested the effects of TUDCA on autophagic dysfunction in obese mice.* Material and Methods.* 500 mg/kg of TUDCA was injected into obese mice, and metabolic parameters, autophagy markers, and insulin signaling molecular were assessed by Western blotting and real-time PCR.* Results.* The TUDCA injections in the obese mice resulted in a reduced body weight gain, lower blood glucose, and improved insulin sensitivity compared with obese mice that were injected with vehicle. Meanwhile, TUDCA treatment not only reversed autophagic dysfunction and endoplasmic reticulum stress, but also improved the impaired insulin signaling in the liver of obese mice. Additionally, the same results obtained with TUDCA were evident in obese mice treated with the adenoviral Atg7.* Conclusions.* We found that TUDCA reversed abnormal autophagy, reduced ER stress, and restored insulin sensitivity in the liver of obese mice and that glycolipid metabolism disorder was also improved via the restoration of defective hepatic autophagy.

## 1. Introduction

Obesity is a causative factor in the development of several pathologies including diabetes and other metabolic diseases, cardiovascular diseases, and cancer [1]. The liver is a major organ regulating glucose and lipid metabolism, and hence it plays a key role in the development of obesity. Nonalcoholic fatty liver disease (NAFLD) is the liver condition most commonly associated with obesity, and it includes a spectrum of liver disorders ranging from steatosis without inflammation to nonalcoholic steatohepatitis, which in turn is a significant cause of more serious diseases such as liver cirrhosis and hepatocellular carcinoma [2, 3]. There is a clear relationship between the degree of obesity and NAFLD prevalence, with this prevalence being greater than 80% in the presence of morbid obesity [4]. However, the exact mechanism underlying liver steatosis remains unknown.

Autophagy is a highly regulated process involved in the turnover of long-lived proteins, cytosolic components, and damaged organelles [5]. Autophagy and endoplasmic reticulum (ER) stress have recently been considered as key regulators of insulin resistance in peripheral tissues, especially in the liver. For example, the levels of autophagy indicators have been found to be markedly decreased in the liver of obese mice, while suppression of autophagy resulted in insulin resistance and ER stress [6]. Consistent with this, Atg7 and Atg5 knockout in hepatocytes resulted in the accumulation of lipid droplets and the activation of ER stress, accompanied by decreased insulin signaling and impaired glucose tolerance, further supporting the associations among abnormal autophagy, activation of ER stress, and insulin resistance in the liver [6]. Several authors have also speculated that autophagy can be beneficial for cells by disposing of damaged cell structures caused by ER stress, whereas that defective autophagy may lead to the failure of restoration of cellular homeostasis, including organelle function [7–9], thus exacerbating insulin resistance and possibly other metabolic pathologies associated with obesity.

Tauroursodeoxycholic acid (TUDCA) is one of the chemical chaperones that constitute a group of low-molecular-weight compounds known to modulate ER function, stabilize protein conformation, improve the folding capacity of the ER, and facilitate the trafficking of mutant proteins [10]. A recent study found that TUDCA could alleviate the increased ER stress seen in obesity and reverse insulin resistance and type 2 diabetes in experimental models [11, 12], suggesting TUDCA as a promising new regulator for mediating autophagy, ER stress, and insulin resistance via certain signaling pathways in the liver of obese mice. However, the intracellular events responsible for TUDCA-mediated effects in autophagy, ER stress, and insulin resistance remain elusive.

The present study provides evidence that TUDCA can reverse abnormal autophagy, reduce ER stress, and restore insulin sensitivity in the liver of the mice fed the high-fat diet. These results support the hypothesis that TUDCA improves the defective hepatic autophagy, activation of ER stress, and impaired insulin signaling induced by obesity, thereby offering novel opportunities for the treatment of obesity.

## 2. Methods

### 2.1. Materials

All chemicals used were of analytical grade and were purchased from Sigma (St. Louis, MO) unless otherwise stated. The following antibodies were used: anti-Atg7, anti-LC3, anti-p-PERK, anti-PERK, anti-p-IR, and anti-IR (Cell Signaling Technology Inc., Danvers, MA); anti-G6Pase, anti-Pck1, anti-p62, anti-p-Akt, anti-Akt, anti-p-eIF2*α*, anti-eIF2*α*, anti-GAPDH, and peroxidase goat anti-rabbit IgG and peroxidase goat anti-mouse IgG from Santa Cruz Biotechnology (Santa Cruz Biotechnology Inc., CA).

### 2.2. Animals Care

This study was carried out in strict accordance with the recommendations in the Guide for the Care and Use of Laboratory Animals of the National Institutes of Health. The protocol was approved by the Committee on the Ethics of Animal Experiments of Medical School of Xi'an Jiaotong University (Permit number: 2014-009). All surgery was performed under sodium pentobarbital anesthesia (40 mg/kg), and all efforts were made to minimize suffering. C57BL/6J mice (4-week-old) were housed under standard conditions with a 12 h light/dark cycle (darkness from 7:30 p.m. to 7:30 a.m.). Mice were distributed into four groups (*n* = 15 per group): (1) vehicle (normal chow diet, 4% of energy as fat, 3.85 kcal/g, plus 10 *μ*L/g of 0.9% NaCl i.p. injection); (2) TUDCA (normal chow plus 500 mg/kg of TUDCA i.p. injection); (3) high-fat + vehicle (diet containing 60% of energy as fat, 5.24 kcal/g, plus 10 *μ*L/g of 0.9% NaCl i.p. injection); (4) high-fat + TUDCA (high-fat diet plus 500 mg/kg of TUDCA i.p. injection). Daily injections of TUDCA or normal saline solution (vehicle) were initiated after mice were fed a high-fat diet for 8 weeks. Mice were injected once a day (6 p.m.) intraperitoneally (i.p.) with 500 mg/kg of TUDCA or with vehicle for a further 8 weeks. Additionally, adenovirus carrying Atg7 or GFP was delivered into the mice which had been fed a high-fat diet for 8 weeks via orbital venous plexus at a titer of 3 × 10^11^ vp/mice for a further 10 days. At the end of the study period, half of mice in each group were randomly selected and received an intraperitoneal injection of insulin at a dosage of 2 IU/kg; 15 minutes after the injection, all mice were euthanized and the liver tissue was obtained and stored at −80°C for subsequent analysis.

### 2.3. Measurement of Serum Hormones and Metabolites

Morning blood glucose and insulin levels were measured as previously described [13].

### 2.4. Metabolic Tests

Glucose tolerance testing (GTT) and insulin tolerance testing (ITT) were performed as previously described [14].

### 2.5. Electron Microscopy Analysis

Superficial gastrocnemius muscles were fixed in 4% paraformaldehyde/2% glutaraldehyde/0.1 M sodium cacodylate pH 7.3, postfixed in 1% osmium tetraoxide, and embedded in epoxy resin (Epon). Ultrathin sections (80 nm) were stained with aqueous uranyl acetate and lead citrate and examined with a JEOL 2000FX transmission electron microscope (JEOL, Peabody, MA). Sixteen electron micrographs per mouse were digitized and the area and number of clearly distinguishable mitochondria were analyzed using Osteomeasure software (OsteoMetrics, Decatur, GA). For quantification of autophagolysosome-like vacuoles, the numbers of autophagolysosomal-like vacuoles were counted in each field and normalized by the surface area.

### 2.6. Liver Histomorphometry

Liver samples (5 × 5 × 5 mm) were fixed in paraformaldehyde 4%/1x PBS, washed three times with 1x PBS, and equilibrated in sucrose 20%/1x PBS, before being embedded in OCT (optimal cutting temperature) compound. Samples were next sectioned at 10 *μ*m using a cryostat. The sections were air-dried, postfixed in formalin, rinsed with 60% isopropanol, stained with Oil Red O (in 60% isopropanol), and counterstained with hematoxylin. The Oil Red O positive area over total area was quantified using Quantity One software.

### 2.7. Gene Expression Analysis

The real-time PCR was applied to DNAseI-treated total RNA converted into cDNA using primers (SuperArray Bioscience, Frederick, MD) and the Taq SYBR Green Supermix with ROX (Bio-rad, Hercules, CA) on a PCR system (MX3000, Agilent Technologies, Santa Clara, CA). *β*-actin amplification was used as an internal reference for each sample.

### 2.8. Western Blotting

Tissues and cells under various treatments were lysed in lysis buffer containing 25 mM Tris HCl (pH 6.8), 2% SDS, 6% glycerol, 1% 2-mercaptoethanol, 2 mM phenylmethylsulfonyl fluoride, 0.2% bromophenol blue, and a protease inhibitor cocktail for 20 min. Western blotting was performed by utilizing a standard protocol as previously described [14].

### 2.9. Statistics

The data was expressed as mean ± SEM in each bar graph. The results were analyzed by two-way ANOVA (two variables), one-way ANOVA followed by Dunnett's* post hoc* test (one variable, more than two groups), or two-tailed Student's *t*-test (two groups). *P* < 0.05 was considered to be significant. Statistical analyses were performed using IBM SPSS 20.0 software.

## 3. Results

### 3.1. Effects of TUDCA on Systemic Glucose Homeostasis and Insulin Sensitivity in Obese Mice

Given the potential therapeutic relevance of TUDCA* in vivo*, we investigated its effects on glucose metabolism and insulin sensitivity in mice with obesity induced by consuming a high-fat diet. The administration of TUDCA was initiated after mice consumed a high-fat diet or a normal diet for 8 weeks. As expected, those mice consuming a high-fat diet had elevated body weight, blood glucose level, and insulin level and developed glucose intolerance and insulin insensitivity as measured by glucose tolerance testing (GTT) and insulin tolerance testing (ITT) (Figures 1(a)–1(g)). The obese mice that were subsequently injected with TUDCA displayed significantly lower body weight, blood glucose level, and serum insulin level and improved glucose tolerance and insulin sensitivity in comparison with the mice consuming the high-fat diet that were injected with vehicle (Figures 1(a)–1(g)). These findings demonstrate that TUDCA exerts positive effects on systemic glucose homeostasis and insulin sensitivity in obese mice.

### 3.2. Effects of TUDCA on Liver Steatosis in Obese Mice

NAFLD is known to be strongly associated with obesity, which is due to the accumulation of lipids in the liver of mice that consume a high-fat diet, which in turn eventually results in the development of liver steatosis [15]. As shown in Figures 2(a)–2(c), the liver of obese mice injected with TUDCA was lighter than that of the mice consuming a high-fat diet that were injected with vehicle, and little lipid accumulation was found in liver sections stained with Oil Red O in the TUDCA-treated obese mice. In addition, the RNA and protein expressions of tumor necrosis factor *α* (TNF*α*), interleukin- (IL-) 6, and IL-8, which are a group of inflammatory factors, were significantly increased in the liver of obese mice but were normalized after injecting TUDCA (Figures 2(d)–2(h)). This indicates that the inflammation typically associated with liver steatosis was absent in the liver of obese mice treated with TUDCA.

### 3.3. Effects of TUDCA on Hepatic Glucose and Lipid Metabolism* In Vivo*

As a major organ regulating glucose and lipid metabolism, the liver plays a key role in the synthesis and degradation (oxidation) of fatty acids [16]. To determine the effects of TUDCA on hepatic glucose homeostasis, we examined the hepatic glycogen content and lipid metabolism of mice. As shown in Figures 3(a)–3(d), the RNA and protein levels of glucose-6-phosphatase (G6pase) and phosphoenolpyruvate carboxykinase 1 (Pck1) were lower in obese mice receiving TUDCA than in the mice consuming the high-fat diet that were injected with vehicle, indicating that TUDCA improved hepatic gluconeogenesis in the obese mice. We therefore also evaluated *β*-oxidation by measuring the release of ^14^CO_2_ after administering [1–14] oleic acid. The *β*-oxidation rate and *β*-oxidation-related genes such as peroxisome proliferator-activated receptor *α* (Ppar*α*) and carnitine palmitoyltransferase 1*α* (Cpt1*α*) were markedly downregulated in mice consuming a high-fat diet, while TUDCA treatment partially restored the expression levels of *β*-oxidation rate and related genes (Ppar*α* and Cpt1*α*) in obese mice (Figures 3(e)–3(g)). In contrast, the expression of lipogenic genes (Fas and Scd1) was upregulated in the liver of obese mice, and those mice injected with TUDCA showed significant downregulation of lipogenic genes compared to the mice consuming the high-fat diet that were injected with vehicle (Figures 3(h) and 3(i)).

### 3.4. Effects of TUDCA on Hepatic Autophagic Response, ER Stress and Insulin Signaling in the Liver of Obese Mice

To determine the role of autophagy and ER stress in the liver of obese mice, we used Western blotting to measure the protein expressions of autophagy and ER stress indicators in the liver. Autophagic indicators such as Atg7 and light chain 3 II (LC3-II) were significantly reduced in the liver of obese mice. In contrast, p62 (also called SQSTM1, which is involved in aggresome formation and degraded through autophagy) [17] was increased in the liver of obese mice compared to mice consuming the normal diet (Figures 4(a) and 4(b)). However, autophagy indicators such as Atg7 and LC3-II were increased significantly while p62 was decreased in the liver of obese mice injected with TUDCA by comparison with obese mice injected with vehicle (Figures 4(a) and 4(b)). Electron microscopy (EM) examinations of the liver demonstrated a slight reduction in autophagosome/autolysosome formation in obese mice by comparison with mice consuming the normal diet, whereas autophagosome/autolysosome formation was elevated in obese mice injected with TUDCA compared to obese mice injected with vehicle (Figures 4(c) and 4(d)), supporting the biochemical alterations in key autophagy molecules. Moreover, we found a significant increase in phosphorylated protein-kinase-like endoplasmic reticulum kinase (PERK) and eukaryotic initiation factor 2*α* (eIF2*α*) in the liver of obese mice, while the liver of the mice consuming the high-fat diet that were injected with TUDCA displayed reduced ER stress, based on the downregulation of phosphorylated PERK and eIF2*α* proteins in comparison to obese mice injected with vehicle (Figures 4(e) and 4(f)).

We next used Western blotting to measure the protein expressions of indicators of insulin receptor signaling. The liver of mice consuming the high-fat diet and injected with vehicle displayed impaired insulin signaling, as evidenced by insulin-stimulated tyrosine 1162/1163 phosphorylation of insulin receptor *β* (IR*β*) subunit and serine 473 phosphorylation of Akt compared with mice that consumed the normal diet (Figures 4(g) and 4(h)). Meanwhile, insulin signaling was restored in the liver of obese mice injected with TUDCA, based on the upregulation of phosphorylated IR*β* and Akt by comparison with obese mice injected with vehicle (Figures 4(g) and 4(h)). This indicates that TUDCA improved glycolipid metabolism disorder partially by recovering the abnormal autophagy and ER stress in the liver of obese mice.

### 3.5. Improvement of ER Stress and Insulin Signaling by the Restoration of Atg7 in the Liver of Obese Mice

To further check whether the defects in hepatic autophagy in obesity are the cause of insulin resistance* in vivo*, we restored Atg7 via an adenoviral system in the liver of obese mice. After delivering the adenovirus, we found that the expression of Atg7 was significantly elevated in the liver tissue of obese mice compared to vector controls, which resulted in increased autophagosome/autolysosome formation and autophagy indicators, as evident by a higher LC3-II and a decreased p62 expression level in the liver. These observations indicated that Atg7 and autophagic activity in the liver of obese mice were restored successfully* in vivo* (Figures 5(a)–5(d)). Meanwhile, restoration of Atg7 expression resulted in a significant reduction in obesity-induced ER stress in the liver of obese mice, as evidenced by decreased levels of phosphorylated PERK and eIF2*α* (Figures 5(e) and 5(f)). Moreover, insulin stimulation in the liver of Atg7-expressing obese mice led to markedly enhanced phosphorylated IR*β* and Akt levels by comparison with controls (Figures 5(g) and 5(h)) and improved glucose tolerance and insulin sensitivity as measured by GTT and ITT (Figures 5(i)–5(l)), indicating that the restoration of Atg7 rescued the defects in insulin receptor signaling and improved glucose homeostasis.

## 4. Discussion

This study has demonstrated that TUDCA can improve glycolipid metabolism disorder in the liver of obese mice via the restoration of defective hepatic autophagy, which causes impaired hepatic insulin sensitivity and glucose homeostasis in obesity. The present results indicate that autophagic dysfunction in the liver may be a relevant mechanism for the two main pathological arms of insulin resistance in obesity: activation of ER stress and impaired insulin signaling. We found that impaired autophagy could contribute to ER stress in obese mice and that the restoration of autophagy via treatment with TUDCA or an adenovirus carrying Atg7 resulted in improvements in ER stress, insulin signaling, and glycolipid metabolism* in vivo*. It is therefore plausible that autophagy can facilitate the elimination or repair of damaged organelles and assist their adaptive responses in restoring metabolic homeostasis. Actually, ER stress can induce autophagy to participate in the degradation of unfolded proteins and in the removal of superfluous ER membranes [18]. ER function could be impaired if this is not achieved, which creates a vicious cycle resulting in metabolic deterioration, insulin resistance, and type 2 diabetes. Future studies should address whether other mechanisms are also involved in the interaction between autophagy and ER stress.

There is a strong relationship between defective autophagy and insulin resistance in obese mice, which has a major effect on glycolipid metabolism. This study has shown that suppressing autophagy not only results in insulin insensitivity, but also influences hepatic gluconeogenesis and *β*-oxidation in obese mice. Consistent with our results, another study showed that suppressing Atg7 expression in the liver tissue of lean mice treated with adenovirus carrying Atg7 shRNA reduced the autophagy deficiency by 80%, in turn resulting in ER stress in the liver tissue of lean mice, as evident by the induction of eIF2*α* and PERK phosphorylation and of Chop, which are three well-known ER stress indicators. Meanwhile, the lean mice treated with adenovirus carrying Atg7 shRNA developed glucose intolerance and insulin insensitivity as measured by GTT and ITT, thereby also demonstrating the importance of autophagy in maintaining glucose homeostasis.

In line with our results, recent studies found that TUDCA administration significantly improved the* in vivo* responses to insulin in ob/ob mice and that the impaired glucose tolerance seen in vehicle-treated ob/ob mice was corrected upon treatment with TUDCA via inhibiting the activation of ER stress and restoring impaired insulin signaling [11, 12]. However, another study found that the effects of an ER protectant on glucose homoeostasis varied in different models of type 2 diabetes: while PBA (a kind of chemical chaperone) normalized hyperglycemia in ob/ob mice, it did not exert a glucose-lowering effect in Goto-Kakizaki rats and had no preventive or therapeutic effects on insulin resistance or hyperglycemia in mice treated with hydrocortisone [19, 20]. Our results also differ from previous findings in elegant experiments involving the foz/foz mice model, wherein ER stress was not a feature associated with insulin resistance and steatohepatitis in the foz/foz model and that altering or protecting ER functions had no effect on insulin resistance and liver disease propagation [21–23]. We therefore consider that at least some of the previous findings could be model-specific. The progressive liver disease of the HFD-fed foz/foz mice—including hepatocellular injury with ballooning, apoptosis, and inflammation and later accompanied by pericellular fibrosis—indicates that this model differs from the diet-induced obese mice model and the ob/ob mice model, inferring that TUDCA may improve liver steatosis in the early stage of NAFLD.

In conclusion, we found that TUDCA reversed abnormal autophagy, reduced ER stress, and restored insulin sensitivity in the liver of obese mice. Additionally, glycolipid metabolism disorder was improved in the liver of obese mice via the restoration of defective hepatic autophagy. The results of this study suggest not only a new concept for the treatment of obesity involving autophagy, but also the novel potential of TUDCA as an effective therapeutic candidate for liver steatosis in the early stage of NAFLD.

## Figures and Tables

**Figure 1:** Effects of TUDCA on systemic glucose homeostasis and insulin sensitivity in obese mice. All analyses were performed in mice fed a normal diet (ND) or a high-fat diet (HFD) for 8 weeks and then injected daily with 500 mg/kg of TUDCA or with vehicle (Veh) for 8 weeks. (a) Body weight. (b) Blood glucose. (c) Serum insulin. (d) Glucose tolerance testing (GTT). (e) Insulin tolerance testing (ITT). (f) Area under the curve by GTT. (g) Area under the curve by ITT. Fifteen mice per group were analyzed. The data was expressed as mean ± SEM in each bar graph. ^*∗*^ *P* < 0.05 (HFD/TUDCA versus HFD/Veh). ^#^ *P* < 0.05 (HFD/Veh versus ND/Veh).

**Figure 2:** Effects of TUDCA on liver steatosis in obese mice. All analyses were performed in mice fed a normal diet (ND) or a high-fat diet (HFD) for 8 weeks and then injected daily with 500 mg/kg of TUDCA or with vehicle (Veh) for 8 weeks. (a) Liver weight. (b) Oil Red O staining of liver sections (magnification 100x). (c) Histomorphometric quantification of the Oil Red O positive area in liver. (d) Relative expression of TNF*α* in liver (real-time PCR). (e) Relative expression of IL-6 in liver (real-time PCR). (f) Relative expression of IL-8 in liver (real-time PCR). (g) Protein expression of TNF*α*, IL-6, and IL-8 in liver. (h) The relative protein quantity of TNF*α*, IL-6, and IL-8 in liver. The relative quantity of proteins was analyzed using Quantity One software. A representative blot is shown and the data was expressed as mean ± SEM in each bar graph. ^*∗*^ *P* < 0.05 (HFD/TUDCA versus HFD/Veh). ^#^ *P* < 0.05 (HFD/Veh versus ND/Veh).

**Figure 3:** Effects of TUDCA on hepatic glucose and lipid metabolism* in vivo*. All analyses were performed in mice fed a normal diet (ND) or a high-fat diet (HFD) for 8 weeks and then injected daily with 500 mg/kg of TUDCA or with vehicle (Veh) for 8 weeks. (a) Relative expression of G6pase in liver (real-time PCR). (b) Relative expression of Pck1 in liver (real-time PCR). (c) Protein expression of G6pase and Pck1 in liver. (d) The relative protein quantity of G6pase and Pck1 in liver. (e) Fatty acid oxidation (pmol/g). (f) Relative expression of Ppar*α* in liver (real-time PCR). (g) Relative expression of Cpt1*α* in liver (real-time PCR). (h) Relative expression of Fas in liver (real-time PCR). (i) Relative expression of Scd1 in liver (real-time PCR). The relative quantity of proteins was analyzed using Quantity One software. A representative blot is shown and the data was expressed as mean ± SEM in each bar graph. ^*∗*^ *P* < 0.05 (HFD/TUDCA versus HFD/Veh). ^#^ *P* < 0.05 (HFD/Veh versus ND/Veh).

**Figure 4:** Effects of TUDCA on hepatic autophagic response, ER stress, and insulin signaling in the liver of obese mice. All analyses were performed in mice fed a normal diet (ND) or a high-fat diet (HFD) for 8 weeks and then injected daily with 500 mg/kg of TUDCA or with vehicle (Veh) for 8 weeks. (a) Protein expression of Atg7, p62, and LC3 in liver. (b) The relative protein quantity of Atg7, p62, and LC3 in liver. (c) Quantification of autophagolysosome-like vacuoles per field in the EM images of liver (magnification 40000x). (d) Quantification of autophagolysosome-like vacuoles per field in the EM images of liver. (e) Phosphorylation of PERK and eIF2*α* in liver. (f) The relative protein quantity of p-PERK and p-eIF2*α* in liver. (g) Phosphorylation of IR and Akt in liver. (h) The relative protein quantity of p-IR and p-Akt in liver. The relative quantity of proteins was analyzed using Quantity One software. A representative blot is shown and the data was expressed as mean ± SEM in each bar graph. ^*∗*^ *P* < 0.05 (HFD/TUDCA versus HFD/Veh). ^#^ *P* < 0.05 (HFD/Veh versus ND/Veh).

**Figure 5:** Improvement of ER stress and insulin signaling by the restoration of Atg7 in liver of obese mice. All analyses were performed in mice fed a high-fat diet (HFD) for 8 weeks and then adenovirus carrying Atg7 or GFP was delivered into obese mice via orbital venous plexus at a titer of 3 × 10^11^ vp/mice. (a) Protein expression of Atg7, p62, and LC3 in liver. (b) The relative protein quantity of Atg7, p62, and LC3 in liver. (c) Quantification of autophagolysosome-like vacuoles per field in the EM images of liver (magnification 40000x). (d) Quantification of autophagolysosome-like vacuoles per field in the EM images of liver. (e) Phosphorylation of PERK and eIF2*α* in liver. (f) The relative protein quantity of p-PERK and p-eIF2*α* in liver. (g) Phosphorylation of IR and Akt in liver. (h) The relative protein quantity of p-IR and p-Akt in liver. (i) GTT. (j) Area under the curve by GTT. (k) ITT. (l) Area under the curve by ITT. The relative quantity of proteins was analyzed using Quantity One software. A representative blot is shown and the data was expressed as mean ± SEM in each bar graph. ^*∗*^ *P* < 0.05 (HFD/Ad-Atg7 versus HFD/Ad-GFP).

## References

[1] Matsuda M., Shimomura I. (2013). Increased oxidative stress in obesity: implications for metabolic syndrome, diabetes, hypertension, dyslipidemia, atherosclerosis, and cancer. *Obesity Research and Clinical Practice*.

[2] de Alwis N. M. W., Day C. P. (2008). Non-alcoholic fatty liver disease: the mist gradually clears. *Journal of Hepatology*.

[3] Baffy G., Brunt E. M., Caldwell S. H. (2012). Hepatocellular carcinoma in non-alcoholic fatty liver disease: an emerging menace. *Journal of Hepatology*.

[4] Lazo M., Hernaez R., Eberhardt M. S. (2013). Prevalence of nonalcoholic fatty liver disease in the United States: the third national health and nutrition examination survey, 1988–1994. *American Journal of Epidemiology*.

[5] Yorimitsu T., Klionsky D. J. (2005). Autophagy: molecular machinery for self-eating. *Cell Death and Differentiation*.

[6] Yang L., Li P., Fu S., Calay E. S., Hotamisligil G. S. (2010). Defective hepatic autophagy in obesity promotes ER stress and causes insulin resistance. *Cell Metabolism*.

[7] Zhang Y., Goldman S., Baerga R., Zhao Y., Komatsu M., Jin S. (2009). Adipose-specific deletion of autophagy-related gene 7 (atg7) in mice reveals a role in adipogenesis. *Proceedings of the National Academy of Sciences of the United States of America*.

[8] Baerga R., Zhang Y., Chen P.-H., Goldman S., Jin S. (2009). Targeted deletion of autophagy-related 5 (atg5) impairs adipogenesis in a cellular model and in mice. *Autophagy*.

[9] Jung H. S., Chung K. W., Won Kim J. (2008). Loss of autophagy diminishes pancreatic beta cell mass and function with resultant hyperglycemia. *Cell Metabolism*.

[10] Xie Q., Khaoustov V. I., Chung C. C. (2002). Effect of tauroursodeoxycholic acid on endoplasmic reticulum stress-induced caspase-12 activation. *Hepatology*.

[11] Özcan U., Cao Q., Yilmaz E. (2004). Endoplasmic reticulum stress links obesity, insulin action, and type 2 diabetes. *Science*.

[12] Özcan U., Yilmaz E., Özcan L. (2006). Chemical chaperones reduce ER stress and restore glucose homeostasis in a mouse model of type 2 diabetes. *Science*.

[13] Zhou B., Li H., Xu L., Zang W., Wu S., Sun H. (2013). Osteocalcin reverses endoplasmic reticulum stress and improves impaired insulin sensitivity secondary to diet-induced obesity through nuclear factor-*κ*B signaling pathway. *Endocrinology*.

[14] Zhou B., Li H., Liu J. (2013). Intermittent injections of osteocalcin reverse autophagic dysfunction and endoplasmic reticulum stress resulting from diet-induced obesity in the vascular tissue via the NF*κ*B-p65-dependent mechanism. *Cell Cycle*.

[15] Anstee Q. M., Goldin R. D. (2006). Mouse models in non-alcoholic fatty liver disease and steatohepatitis research. *International Journal of Experimental Pathology*.

[16] Tilg H., Moschen A. R. (2008). Insulin resistance, inflammation, and non-alcoholic fatty liver disease. *Trends in Endocrinology and Metabolism*.

[17] Bjørkøy G., Lamark T., Brech A. (2005). p62/SQSTM1 forms protein aggregates degraded by autophagy and has a protective effect on huntingtin-induced cell death. *The Journal of Cell Biology*.

[18] Bernales S., Schuck S., Walter P. (2007). ER-phagy: selective autophagy of the endoplasmic reticulum. *Autophagy*.

[19] Xu T.-Y., Chen R.-H., Wang P., Zhang R.-Y., Ke S.-F., Miao C.-Y. (2010). 4-Phenyl butyric acid does not generally reduce glucose levels in rodent models of diabetes. *Clinical and Experimental Pharmacology and Physiology*.

[20] Rinella M. E., Siddiqui M. S., Gardikiotes K., Gottstein J., Elias M., Green R. M. (2011). Dysregulation of the unfolded protein response in db/db mice with diet-induced steatohepatitis. *Hepatology*.

[21] Legry V., Van Rooyen D. M., Lambert B. (2014). Endoplasmic reticulum stress does not contribute to steatohepatitis in obese and insulin-resistant high-fat-diet-fed foz/foz mice. *Clinical Science*.

[22] Wu S.-D., Li L., Wang J.-Y. (2012). Ursodeoxycholic acid for nonalcoholic steatohepatitis. *European Journal of Gastroenterology and Hepatology*.

[23] Dara L., Ji C., Kaplowitz N. (2011). The contribution of endoplasmic reticulum stress to liver diseases. *Hepatology*.

